# Effect of Ultrasound Image-Guided Nerve Block on the Postoperative Recovery Quality of Patients with Tibial Fractures Using the Concept of Enhanced Recovery after Surgery

**DOI:** 10.1155/2022/4428883

**Published:** 2022-08-22

**Authors:** Xiaohong Zhang, Lu He, Xiangqing Mo, Ling Jiang, Chenhui Deng

**Affiliations:** Department of Postanesthesia Care Unit (PACU), Zhuzhou Central Hospital, Zhuzhou, 412000 Hunan, China

## Abstract

This study was aimed at investigating the clinical effect of ultrasound-guided nerve block based on the concept of enhanced recovery after surgery (ERAS) for postoperative anesthesia in patients with tibial fractures. The noise-reduction processing was introduced in ultrasound images to adjust the ultrasound clarity of the patient. A total of 177 patients with tibial fractures in our hospital were retrospectively analyzed and divided into OG group (general anesthesia combined with nerve block, 78 cases), C1 group (simple general anesthesia, 27 cases), C2 group (ultrasound-guided nerve block combined with general anesthesia, 10 cases), and C3 group (62 cases of spinal-epidural anesthesia). The effect of anesthesia and postoperative recovery time of patients in each group were analyzed. The wake-up time of the OG group was significantly shorter than that of the other three groups (*P* < 0.05). The doses of propofol and remifentanil in the OG group were much lower than those in the other groups (*P* < 0.05). After the ultrasound image was processed with noise reduction, the image showed the lesion more clearly. The excellent and good rates of OG group, C1 group, C2 group, and C3 group were 89.86%, 62.73%, 75.37%, and 61.07%, respectively. The Ramsay sedation score and anesthesia satisfaction in the OG group were obviously higher than those in the other groups, but there was no significant difference (*P* > 0.05). The visual analogue scale (VAS) scores of the OG group at 12 h, 24 h, and 36 h after the surgery were 4.52 ± 0.41, 4.72 ± 0.24, and 4.81 ± 0.74, respectively, which were significantly higher than those of the other three groups (*P* < 0.05). On the basis of ERAS, ultrasound-guided nerve block combined with general anesthesia can improve the perioperative pain in patients with tibial fractures and significantly shorten the time for the wake-up time. In addition, it was safe and reliable, so it was worthy of clinical promotion.

## 1. Introduction

The tibia and fibula are located under the human skin without muscle covering, which is a common type of long bone fractures in patients with orthopedic fractures. In recent years, the incidence has been rising, and after fracture, the skin is easily pierced by the fracture end, which can lead to traumatic arthritis over time [1]. Due to the damage of external force, the soft tissue can easily cause serious damage, which has a great impact on the health and quality of life of patients [2, 3]. Surgery is an important modality for the treatment of tibial fractures, and ensuring the safety and effectiveness of anesthesia is a very important feature. Studies have shown that nerve block anesthesia combined with general anesthesia can effectively improve myocardial oxygenation, showing a good anesthesia effect, especially for patients with underlying cardiovascular diseases [4]. The methods of intraoperative anesthesia include central nerve axon block (spinal, epidural or combined spinal-epidural block), lumbar plexus nerve block with posterior approach block (psoas compartment block), and anterior approach block (parainguinal block). Different anesthesia methods vary in terms of postoperative analgesia, type of surgery, rehabilitation, and patient satisfaction [5]. Capdevila et al. [6] showed that persistent peripheral nerve block is an effective analgesic technique for postoperative sedation of orthopedic pain, and neurological and infectious adverse events are rare. The postoperative analgesic effect of regional nerve block is better than systemic administration of morphine, and the adverse reactions are also less than epidural anesthesia. The previous nerve blocks were all difficult to operate, and they all located the target nerve by blind detection, which could not confirm the diffusion range of anesthesia and could not guarantee the effect of the block. Even if the anesthesiologist has rich experience, there will be anatomical variations, individual differences, and other factors that may lead to inaccurate injection of anesthesia drugs and poor nerve block results [7, 8]. With the continuous development of medical technology, ultrasound-guided nerve block technology has been widely used in clinical practice. Ultrasound can visualize the positioning of nerves, accurately inject anesthetic doses, and effectively avoid damage to blood vessels and nerves, and patients do not need to change their positions. After systemic induction, the pain of patients is greatly reduced [9]. The nerve block operation under ultrasound-guided is simple and accurate, and the patient can be extubated as soon as possible after waking up. Using ultrasound-guided can not only clearly display the patient's spinal anatomy but also observe the patient's anatomical condition before puncture in real time, making it easier for physicians to understand the surgical process, ensuring the safety of the nerve block, and greatly improving the success rate of the operation [10–12].

The middle and lower third of the tibia is prone to fracture, the lower end of the calf is compressed, and severe avascular necrosis occurs. The concept of enhanced recovery surgery for the middle and lower tibia originated from cardiac surgery, and now it has been extended to vascular surgery, plastic surgery, colorectal surgery, joint surgery, hernia surgery, etc. Academician Li Jieshou's team has shown in the study of gastric cancer patients that the treatment of this concept is safe and effective [13, 14]. Anesthesia methods in the enhanced recovery surgery concept include general anesthesia, regional block, and a combination of the two. Such anesthesia method can not only meet the basic requirements of sedation, analgesia, and improve good surgical adjustment but also effectively reduce the surgical stress, which is beneficial to the postoperative recovery of patients [15]. Enhanced recovery after surgery (ERAS) refers to the clinical scientific practice of patients during the perioperative period, and evidence-based medicine has proven to be an effective measure. ERAS has been integrated into the care of many surgical diseases [16]. Nursing staff use this optimized nursing and monitoring measures to speed up the recovery of patients, shorten the hospitalization time of patients, effectively improve the patient's negative psychology, improve patient satisfaction, and have a positive impact on the incidence of postoperative complications and readmissions [17, 18]. Broadbent et al. [19] stated that it is feasible not to do routine bowel preparation before elective ERAS surgery, and it is not associated with postoperative complications.

This study investigated the effect of ultrasound image-guided nerve block on the resuscitation quality of anesthesia and resuscitation room after tibia surgery under the guidance of ERAS concept. Visualization of ultrasound-guided nerve blocks greatly improved the success rate of nerve blocks. This study could provide a reference for the functional evaluation of patients, shorten the postoperative recovery time of patients, and analyze the anesthesia effect of ultrasound combined with nerve block on patients with tibial fracture.

## 2. Materials and Methods

### 2.1. Research Objects

There were 760 tibial fracture operations performed in 5 years from January 2017 to December 2021, and 177 patients who met the criteria of this study were selected. Among the causes of fracture, there were 66 patients with tibial fracture due to traffic accidents, 47 patients with drops, and 64 patients with falls. The patients were grouped according to the surgical method, 78 cases with general anesthesia and nerve block were OG group, 27 cases with general anesthesia (without nerve block) were group C1, 10 cases with spinal-epidural joint and nerve block were group C2, and 62 cases with spine-epidural anesthesia (without nerve block) were group C3. This study was approved by ethics committee of hospital, and the patients and their families were informed about the study and signed the informed consent.

Inclusion criteria are as follows: patient with tibial fracture on ultrasound; patients with complete clinical data; patients whose American Society of Anesthesiologists (ASA) grade was I-II; patients who were determined as tibial fracture according to the trauma history, clinical symptoms, and examination results; patients with no contraindication to surgical anesthesia; patients with no senile dementia and able to actively cooperate with medical staff in rehabilitation training; and patients not taking glucocorticoids in the past 2 months.

Exclusion criteria are as follows: those who were allergic to the anesthetics; those who were in critical condition and unable to cooperate with the investigator; patients with contraindications; patients with coagulation dysfunction; patients with systemic infection; patients with severe cardiovascular disease or abnormal liver and kidney function; and patients with old fractures.

### 2.2. Fast Track Surgery

Fast track surgery speeded up patient recovery and shortened surgical hospital stays. The measures used in this study to speed up recovery include the following aspects. First, it should talk with the patient before surgery, inform the patient of the surgery plan, obtain the patient's cooperation, and reduce psychological stress. Secondly, it should provide nutritional support before surgery to avoid prolonged application, oral laxatives for bowel preparation and diet control, and 250-400 mL of 10% glucose solution 2 hours before surgery. Thirdly, it should not routinely use the nasogastric tube, urinary catheter, and drainage. Fourthly, it should actively adopt minimally invasive techniques. Fifthly, it should use sedatives and pain relievers before surgery and place an epidural tube for pain relief 1-2 days before surgery. Sixthly, it can choose a reasonable anesthesia method plus general anesthesia. Finally, it can get out of bed in the early stage before surgery and get out of bed for 6-8 hours after surgery. In addition, it should ensure the intraoperative fluid infusion, strictly control infusion volume and infusion speed, and pay attention to the intraoperative thermal insulation to adjust the room temperature to 25°C.

### 2.3. Research Methods

Color ultrasound scanner and high-frequency ultrasound probe were used for ultrasound-guided. After the patient entered the room, electrocardiograph (ECG) monitoring was performed. The venous access was opened, and anesthesia was used for induction. Anesthesia induction was propofol 2.0 mg/kg + fentanyl 3 *μ*g/kg + vecuronium bromide 0.6 mg/kg + midazolam 0.03 mg/kg. When the patient did not lose consciousness and had no blinking reflex, an endotracheal intubation was adopted and connected to a ventilator for mechanical ventilation. Gastrointestinal anesthesia included remifentanil, the drip rate was kept at 0.1 *μ*g/(kg min), combined with intravenous infusion of propofol 3-10 mg/kg, the drip rate was maintained at 4-8 mg/(kg h), and it was stopped 10 minutes before the completion of the surgery.

For the sciatic nerve block, the patient took the affected limb to elevate, the skin was routinely disinfected at the popliteal fossa, and the ultrasound probe was placed between the biceps femoris and the semitendinosus at the proximal 7 cm of the popliteal crease. The sciatic nerve was located using an ultrasound probe and fixed to its distal bifurcation and injected with 0.375% 20 mL ropivacaine.

For the femoral nerve block, the patient was placed in the supine position, routine disinfection was performed in the groin area, and an ultrasound probe was used to place the femoral artery pulse below the inguinal ligament. According to the ultrasound-guided images, the guide needle was inserted in parallel, there was a clear sense of breakthrough, and 0.5% 10 mL ropivacaine was used for the block.

For the observation group (*n* = 78) (OG group), on the basis of general anesthesia and nerve block after induction of anesthesia, the femoral and sciatic nerves were found with the aid of ultrasound.

For the control group 1 (*n* = 27, C1 group), general anesthesia (without nerve block) and the anesthesia method were the same as that of OG group.

For the control group 2 (*n* = 10, C2 group), spinal-epidural anesthesia and nerve block anesthesia, after the patients entered the operating room, peripheral venous access was established, vital signs were detected, and oxygen inhalation nursing was given. The healthy side lying position was selected, and L1-2/L2-3 intervertebral space was determined as the puncture site. Then, it should implant an epidural catheter and inject ropivacaine hydrochloride injection (1.5-2.5 mL 5% ropivacaine after cerebrospinal fluid reflux). Surgery was performed after observing for a few minutes.

For the control group 3 (*n* = 62, C3 group), spine-epidural anesthesia, there was no nerve blocking.

During the surgery, the anesthesia level was adjusted according to the actual situation of the patient, and the dosage of anesthesia was increased according to the actual situation of the patient.

### 2.4. Evaluation Indicators

The related indicators of anesthesia in each group were compared, including recovery time, extubation time, dosage of propofol, and dosage of remifentanil, and the Ramsay sedation score 10 minutes after cupping and the pain degree half an hour after extubation were compared in each group. The visual analogue scale was used to assess the degree of pain. The higher the Ramsay sedation score, the better the effect of sedation. When the score was 0, the higher the score, and the more intense the pain. The VAS score is shown in Table 1.

The adverse reactions in each group were observed, whether the patients had vomiting, nausea, dyspnea, chills, restlessness, and other adverse reactions. According to the effect of anesthesia experienced by the patient, there was no pain, irritability, or discomfort during the operation and no obvious adverse reactions. There was no obvious fluctuation in the intraoperative detection, indicating that the anesthesia was effective, mild pain, discomfort, and irritability during the surgery and no obvious adverse reactions. There was no significant fluctuation in the intraoperative detection indicators, indicating that anesthesia was ineffective.

### 2.5. Statistical Methods

All data in this study were established in Excel database and analyzed using the SPSS 19.0 statistical software. Measurement data were tested by *t* test, and the difference was statistically significant at *P* < 0.05. The enumeration data were analyzed by *χ*^2^ test, and the enumeration data were expressed as percentage (%). It was suggested to compare the effect of anesthesia in each group by using Diehe. According to the grade data of anesthesia effect, the difference was significant at *P* < 0.05.

## 3. Results

### 3.1. Analysis of the Causes of Fractures

In this study, 177 patients who met the criteria of this study were selected. Among the causes of fracture, 66 patients suffered from tibial fracture due to traffic accident, 47 patients dropped, and 64 patients fell. Of the 78 patients in the OG group, 29 patients suffered from tibial fracture due to traffic accidents, accounting for 37.18%; 17 patients suffered from drop injury, accounting for 28.81%; and 32 patients fell, accounting for 54.24%. In the C1 group of 27 patients, 11 patients suffered tibial fracture due to traffic accidents, accounting for 40.74%; 9 patients dropped, accounting for 33.33%; and 7 patients fell, accounting for 25.93%. Among the 10 patients in group C2, 3 patients suffered tibial fracture due to traffic accident, accounting for 30%; 2 patients suffered from drop injury, accounting for 20%; and 5 patients fell, accounting for 50%. Among the 62 patients in the C3 group, 23 patients suffered from tibial fracture due to traffic accidents, accounting for 37.10%; 19 patients dropped, accounting for 30.65%; and 20 patients fell, accounting for 32.26%. There was no statistical difference among the groups (*P* > 0.05). The results are shown in Figure 1.

### 3.2. Analysis of Wake-Up Time

The wake-up time in different groups was compared, and the results are shown in Figure 2. The wake-up time of the OG group was significantly less than the other three groups. There was no significant difference in wake-up time between C1 and C2 groups (*P* > 0.05).

### 3.3. Comparison of Anesthesia Indicators

Figure 3 analyzes the dosage of propofol and remifentanil in each group, which showed that the dosage of the observation group was significantly less than that of the other groups, and the difference was significant (*P* < 0.05). Regarding the dosage of remifentanil, there was a significant difference between the C1 and C2 groups and the C3 group (*P* < 0.05). Propofol dosage showed the same trend. The results are shown in Figure 3.

### 3.4. Comparison of Excellent and Good Rates

The excellent and good rate was 89.86% in the observation group, 62.73% in the C1 group, 75.37% in the C2 group, and 61.07% in the C3 group. The effect of the observation group was significantly higher than that of the other three groups. The specific results are shown in Figure 4.

### 3.5. Postoperative VAS Scores

The VAS scores after 12 h, 24 h, and 36 h in the OG group were 4.52 ± 0.41, 4.72 ± 0.24, and 4.81 ± 0.74, respectively. The VAS scores of C1 group after 12 h, 24 h, and 36 h after surgery were 2.21 ± 0.81, 3.42 ± 0.94, and 3.63 ± 0.76, respectively. The postoperative VAS scores of C2 group after 12 h, 24 h, and 36 h were 4.31 ± 1.78, 4.51 ± 0.94, and 4.62 ± 0.93, respectively; and those in the C3 group were 3.08 ± 1.42, 3.87 ± 0.95, and 3.96 ± 0.69, respectively. Compared with other groups, the OG group had significant difference (*P* < 0.05). The results are illustrated in Figure 5.

### 3.6. Ultrasound Images

Figure 6(a) is an image of the sciatic nerve displayed by ultrasound, and the gray arrow indicated the position of the femoral nerve. The orange arrow in Figure 6(b) shows the femoral nerve and the femoral artery.  Figure 6(c) shows the bevel of the ultrasound-guided tip indicated by the grey arrow.

### 3.7. Comparisons of the Ramsay Sedation Score and Anesthesia Satisfaction

The Ramsay sedation score and anesthesia satisfaction of the OG group were significantly higher than those of the other groups, and there was no significant difference between the OG group and the C2 group (*P* > 0.05). There was significant difference between OG group and C1 and C3 groups (*P* < 0.05). The results are shown in Table 2.

### 3.8. Comparison of Adverse Reactions

Nausea and vomiting occurred in 1.28% of the OG group. Nausea and vomiting occurred in 2 cases in the C1 group, accounting for 7.41%; chills occurred in 1 case, accounting for 3.70%, and agitation occurred in 1 case, accounting for 3.70%. There were 2 cases of nausea and vomiting in group C2, accounting for 20%, 1 case of chills in group C3, accounting for 1.61%, and 2 cases of agitation, accounting for 3.23%. The overall incidence of adverse reactions was 1 in OG, 5 in C1, 2 in C2, and 4 in C3. The observation group had the least number of patients with adverse reactions. The results are shown in Table 3.

## 4. Discussion

For patients in the perioperative period, it is necessary to perfuse both the occurrence of complications (airway obstruction, vomiting, pain, and unstable circulatory function, etc.) and the anesthesia recovery period [20]. As stated in the ERAS application guidelines, the anesthesia management should be optimized as much as possible, and short-acting anesthetics should be selected as much as possible [21]. Postoperative muscle relaxants and anesthetics have not been excreted from the body late, and the reflex phenomenon has not fully recovered. Optimizing nursing care in the recovery room can effectively avoid the occurrence of complications and promote the safety of patients through the perioperative period. ERAS advocates postoperative multimodal analgesia management, including intravenous docaine, intravenous patient-controlled analgesia management, and nonsteroidal anti-inflammatory drugs. Cheng et al. [22] proved that ultrasound-guided lower thoracic paravertebral block under the guidance of ERAS-accelerated surgery concept can provide perfect postoperative analgesia for female percutaneous nephrolithotomy, provide patients with satisfactory anesthesia and postoperative analgesia, and shorten the postoperative recovery time of patients. In the clinical nursing of postoperative resuscitation of patients with general anesthesia in the anesthesia recovery room, it is necessary to closely perfuse the patient's nervous system, respiratory system, digestive system, and circulatory system to improve symptoms and improve prognosis. In this study, 2 patients with general anesthesia had severe nausea and vomiting and arrhythmia, and 2 patients needed to be returned to the intensive care unit in time. 1 patient in the C3 group had chills, and 2 patients had agitation. The overall incidence of adverse reactions was observed, and the number of patients with adverse reactions in the observation OG group was the least. Only 1 case of vomiting occurred, and the rest of the patients recovered smoothly. Effective nursing of patients with general anesthesia in the anesthesia recovery room can promote the safe and early recovery of patients. The nerve block is performed under ultrasound-guided, and there is no need to explore the patient's muscle twitches during the operation.

This surgery is performed in real time after induction of general anesthesia, which avoids the aggravation of pain, reduces the pain of puncture, and helps the patient to eliminate fear. Ultrasound-guided subregional nerve block anesthesia combined with spine-epidural anesthesia has a good effect. During the surgery, the emergency response of the patient's body is inhibited, the myocardial oxygenation of the patient is inhibited, and the unstable cardiac pain and other diseases will be reduced, which is beneficial to related complications such as pulmonary infection. Zhao et al. [23] pointed that ultrasound-guided nerve block anesthesia surgery can effectively improve the intraoperative anesthesia effect of patients with tibial fractures and improve the stability of intraoperative and postoperative hemodynamic indicators. Anesthesia surgery will play a positive role in postoperative pain control, reduce the risk of postoperative adverse reactions, and reduce the activity of inflammatory factors in postoperative patients. This study yielded the same effect. Zhen et al. [24] thought ultrasound-guided paravertebral nerve block anesthesia improved stress and hemodynamic responses in lung cancer thoracic surgery patients without an increase in the incidence of adverse events. Fan et al. [25] used the artificial intelligence algorithm to guide the nerve block by ultrasound images combined with general anesthesia and showed a good effect during the operation. The CNN algorithm can accurately segment the lesions in the ultrasound images of gastric cancer, which is convenient for doctors to make more accurate judgments on the lesions to provide the basis for the preoperative examination of radical gastrectomy for gastric cancer. Ultrasound-guided nerve block combined with general anesthesia can effectively improve the analgesic effect of radical gastrectomy for gastric cancer, can reduce intraoperative and postoperative adverse reactions and the dosage of analgesic drugs, and has a good effect on postoperative recovery of patients. In this study, intelligent noise-reduction processing was implemented in ultrasonic imaging, and the resulting ultrasonic images were clearer. This study showed that the effect was better than that of general anesthesia without nerve block, and the difference was significant (*P* < 0.05). The effect of spinal-epidural anesthesia and nerve block anesthesia was better than spine-epidural anesthesia (without nerve block), and the difference was significant (*P* < 0.05). Ultrasound-guided block combined with spine-epidural anesthesia can avoid the adverse consequences of intraoperative regional nerve block insufficiency.

In anesthesia, the dose of drugs used in anesthesia can be reduced, which is beneficial to the stabilization of the hemodynamic indexes of patients during surgery. The VAS scores of patients with general anesthesia and nerve block were significantly higher than those of the other three groups on the basis of anesthesia induction (*P* < 0.05). It indicated that the degree of pain in all patients decreased after surgery, and the score was the highest at 36 hours after the surgery. This further confirms that the combined anesthesia regimen under ultrasound-guided is more beneficial to improve the quality of surgical anesthesia in patients with tibial fracture.

## 5. Conclusion

Based on the concept of ERAS, this study adopted ultrasound-guided nerve block to analyze the postoperative anesthesia effect of patients with tibial fracture. In patients with tibia, ultrasound-guided nerve block combined with general anesthesia can ensure the effect of anesthesia, reduce the application of anesthesia dose, and improve the safety of anesthesia. The use of ERAS nursing after surgery can effectively guarantee the postoperative effect of patients, which can not only reduce the emergency response of patients but also shorten the extubation time and wake-up time. There were certain shortcomings in this study. Due to the limitation of research time and the lack of long-term follow-up of patients, long-term follow-up of patients was required in the later stage to further verify the long-term efficacy. Next, different anesthesia methods can be compared by analyzing the patient's hemodynamic indicators. It was believed that in the future, clinical applications would have better anesthesia effects for the treatment of tibial fractures.

## Figures and Tables

**Figure 1:** Analysis of the causes of fractures in four groups. OG: OG group; C1: C1 group; C2: C2 group; and C3: C3 group.

**Figure 2:** Comparison results of wake-up time in each group. OG: OG group; C1: C1 group; C2: C2 group; and C3: C3 group.

**Figure 3:** Comparison results of anesthesia-related indicators in each group. OG: OG group; C1: C1 group; C2: C2 group; and C3: C3 group. ^∗^Compared with the other three groups, *P* < 0.05; ^#^compared with the C3 group, *P* < 0.05.

**Figure 4:** Comparison of excellent and good rates in each group. OG: OG group; C1: C1 group; C2: C2 group; and C3: C3 group.

**Figure 5:** VAS scores of each group at different time periods after the surgery. OG: OG group; C1: C1 group; C2: C2 group; and C3: C3 group.

**Figure 6:** Ultrasound images. (a) Ultrasound display of the sciatic nerve; (b) ultrasound display of the femoral artery; (c) ultrasound-guided tip oblique view. The yellow arrows in the figure indicate sciatic nerve and popliteal artery, and the yellow line is puncture bevel.

**Table 1:** VAS score.

Level	Symptoms
0 points	No pain
3 points or less	Tolerable mild pain
4-6 points	Pain interfering with sleep, but can be tolerated
7-10 points	Intense pain that was difficult to bear

**Table 2:** Comparisons of the Ramsay sedation score and anesthesia satisfaction.

Group	Cases	Ramsay sedation score	Anesthesia satisfaction score
OG	78	2.34 ± 0.71	7.81 ± 1.02
C1	27	1.96 ± 0.42	7.02 ± 0.17
C2	10	2.31 ± 0.63	6.73 ± 0.34
C3	62	2.01 ± 0.27	6.21 ± 0.28
*χ* ^2^		2.71	1.013
*P*		0.018	0.429

**Table 3:** Comparison of adverse reactions.

Group	Cases	Nausea and vomiting	Chill	Agitation	Difficulty breathing
OG	78	1	0	0	0
C1	27	2	1	1	0
C2	10	2	0	0	0
C3	62	0	1	2	1
*χ* ^2^		0.476	1.087	1.375	
*P*		0.608	0.387	0.416	

## Data Availability

The data used to support the findings of this study are available from the corresponding author upon request.
